# Facing SARS-CoV-2 outbreak in immunotherapy era

**DOI:** 10.2217/fon-2020-0340

**Published:** 2020-05-29

**Authors:** Fabrizio Citarella, Marco Russano, Francesco Pantano, Emanuela Dell'Aquila, Bruno Vincenzi, Giuseppe Tonini, Daniele Santini

**Affiliations:** ^1^Department of Medical Oncology, Campus Bio-Medico University, Via Alvaro del Portillo 200, Rome 00128, Italy

**Keywords:** COVID-19, immune checkpoint inhibitors, immunotherapy, inflammation, SARS-CoV-2

## Abstract

Severe acute respiratory syndrome coronavirus 2 (SARS-CoV-2) spread represents a sanitary emergency all over the world. Viral biology is only partially known with some aspects in common with other CoV and the damage observed in most severe cases is due to intense inflammation. Immunotherapy restores immunological activity against cancer cells and it has become a standard treatment for several cancers. We carried out an examination of available data concerning with the effects exerted by both SARS-CoV-2 and the most widespread immunotherapy treatments on the immune system in order to hypothesize mechanisms underlying potential and mutual interaction. We provided an analysis of laboratory, clinical and therapeutic data related with severe acute respiratory syndrome coronavirus. We finally focused on implications of immunotherapy treatments in clinical practice.

Since December 2019, the world is facing the rising emergency of novel coronavirus SARS-CoV-2 spread and the severe acute respiratory syndrome coronavirus disease 19 (COVID-19) has become a challenge for global healthcare. With a regeneration number (R0) is 2.2 [1], many countries are being forced to introduce strict limitations in order to reduce risk of contagion and COVID-19 is considered pandemic since 11 March 2020 [2].

At the same time, most of infected people do not report any symptoms, thus prevalence of infection is largely underrated.

Taking into analysis immunological aspects of SARS-CoV-2 infection and effects exerted by immune checkpoints inhibitors (ICI) on immune system, the present work aims at investigating potential implications of viral spread for patients receiving immunotherapy treatment at risk of developing immune related events (irAE). Particular attention is reserved to pneumonitis, since COVID-19 is characterized by prominent lung inflammation; similarly, ICI are able to induce pulmonary immune-mediated inflammation, a condition requiring differential diagnosis. We provide biological insights on viral and ICI effects on immune system and explanations of possible synergistic effects between immunotherapy treatment and SARS-CoV-2-related inflammation.

## The effects of virus on immune system

CoV are single-stranded RNA viruses ranging from 26 to 32 kilobases, being largest RNA genome provided viruses.

α- and β-CoV are responsible for human infections, varying from asymptomatic status until severe pneumonia, acute respiratory syndrome and organ injury. Since both innate and adaptive immune response are involved in limiting infection [3], a significant inflammatory reaction is observed in severe cases.

COVID-19 has been occurring more in non young men patients, often affected by comorbidities; prevalence of malignancy among infected patients was up to 7% in a large report [4]. We can rely on a few instruments to evaluate severity of infection: lymphopenia, higher blood cell count and higher neutrophil count, in association with non specific markers, such as lower albumin, higher prothrombin time and higher D-Dimer, commonly altered in cancer patients, are predictors of poorer outcome during COVID-19 [5,6].

To date, knowledge about interplay between SARS-CoV2 and immune system is only partial; as it shares about 80% of genome sequence with the recent SARS-CoV [7], a few common immunological pathways have been postulated. The binding with angiotensin-converting enzyme 2 allows the virus to infect alveolar epithelial cells, vascular endothelial cells and macrophages and to replicate [7,8].

Immune response includes several mechanisms and some of them are worthy of being enlightened (Table 1):

- Significant increase in inflammatory cytokines occurs in the first phase (such as, IL-7, IL-8, IL-10, monocyte chemoattractant protein-1, TNF-α, IFN-γ) [6].
- SARS-CoV2 Viroporin 3a is able to activate NLRP3 inflammasome paving the way to pyroptosis [9]. Lymphocytes are suspected to be most hit by pyroptosis, thus explaining recurrent lymphopenia [10].
- Complement activation can be induced by SARS-CoV2 contributing to macrophages activation [11].
- After the binding between pathogen-associated molecular patterns and pattern recognition receptors, caspase-1 is activated and damage-associated molecular patterns are released further enhancing inflammation.
- Reduction of ACE2 function by SARS-CoV [12,13] results in lung injury [14,15]; in addition, shedding of ACE2 ectodomain, favored by SARS-CoV [16,17], acts as an inducer of TNF-α [18]. Similar mechanisms are plausible also for SARS-CoV-2, due to sharing of same receptor.
- The viral spike protein is the site of receptor binding and membrane fusion [19] and represents one of the main CoV antigen recognized by humoral and cellular immunity [20]. Antibodies (Ab) against SARS-CoV spike (S) glycoprotein (anti-S-IgG) production is a landmark of pulmonary CoV infection. Similarly to what was observed in patients affected from SARS-CoV [21,22], animal experiments demonstrated that high anti-S-IgG titer, despite suppressing viral replication, is associated with more severe lung injury [23]. Anti-S-IgG Ab could trigger macrophages activation trough Fc receptors, whose inhibition reduces inflammatory storm. Activation of complement and antibody-dependent cell-mediated cytotoxicity are likely induced by anti-S-IgG Ab.
- Macrophages are mainly involved in acute respiratory distress syndrome both in the inflammatory damage and in tissue repairing [24], depending on main acquired polarization, respectively M1 (classical activation) pro-inflammatory or M2 (alternative activation) inflammatory-resolving phenotype [25]. Persistence of inflammation is likely to keep macrophages activation and to interfere with tissue restoring during CoV-induced SARS [26]. Anti-S-IgG Ab promote M2 phenotype acquiring trough TGF-β suppression and IL-8 and monocyte chemoattractant protein-1 induction [23].
- Similarly to SARS [27], outcome of older patients is usually worse than younger during SARS-CoV-2 infection. The entity and severity of infection appears to be influenced by antibody dependent enhancement: presence of anti-S-Ab due to previous exposition to CoV is associated with easier infection from certain other CoV, above all from those with lower affinity for ACE-2 [28]. Many CoV might have circulated in the Chinese population [29], while SARS-CoV should not be considered a significant contributing agent according to sero-prevalence studies [30].
- Both CD4^+^ and CD8^+^ T cells are recruited throughout β-CoV infection. T_reg_ are involved in viral immune contrast, even though their activation delays viral clearance [31]. CD8^+^ T cells represent up to 80% of cells involved in lung inflammation during SARS assuring viral clearing but also causing inflammatory damage. However, CD4^+^ T cells promote lymphocytes recruitment and antibodies and cytokines production; their deficiency *in vivo* results in more severe immune-pulmonary infection and delayed viral clearance during SARS [32].

**Table 1.** Virus effects on inflammatory receptors and mediators.

Receptor and mediators	Effects on immune system	Ref.
ACE 2	Virus receptor leading to target cells infection and lung injury worsening. Shedding of ACE 2 ectodomain increases TNF-α.	[12–18]
Cytokines (IL-7, IL-8, IL-10, MCP-1, TNF-α, IFN-γ)	Inflammatory storm due to immune response to virus invasion	[6]
NLRP3 inflammasome	Pyroptosis induction, involving mostly lymphocytes	[9,10]
Complement	Activation due to virus spread and further macrophages recruitment	[11]
Humoral immunity	Hyperproduction of immunoglobulins accounts for anti-S-protein-IgG, linked both with precocious viral clearance and with worse lung injury	[19–23]
Macrophages	Virus induces macrophages recruitment and M2 polarization with subsequent more severe inflammation	[23–27]
T_reg_	T_reg_ activation delays viral clearance	[31]
CD4^+^ and CD8^+^	Intense recruitment involved in containing virus and consequential pulmonary inflammation	[32]

ACE 2: Angiotensin-converting enzyme 2; MCP-1: Monocyte chemoattractant protein-1.

In summary, the first phase of COVID-19 is driven by viral entrance and invasion, inflammatory stimuli, intense apoptosis and pyroptosis, and complement activation. IL-1 and IL-6 appear to be the most involved inflammatory mediators [33]. Most of patients are able to clear viral infection without reporting any symptom.

Massive neutralizing antibodies arising, whose function is inhibiting viral spread, characterizes the second phase, but they can trigger or exacerbate lung injury. Even though T cells are crucial to control and suppress viral spread, they can exacerbate inflammatory events and CD8^+^ T cells are the main phenotype detectable. Previous exposition to CoV may account for more severe lung damage, thus explaining greater damage observed in older patients.

SARS-CoV-2 related damage is mainly inflammation mediated. Most severe COVID-19 cases are likely to reflect a cytokine storm syndrome leading to worse prognosis [34].

A mirroring example of inflammation is provided by a Chinese report of autopsy carried on three patients dead for COVID-19 [35]. Alveolar damage displayed hyaline membrane formation with a strong infiltration from macrophages and monocytes. Multinucleated giant cells, minimal lymphocytes, eosinophils neutrophils and Type II alveolar cells proliferation and desquamation were also found. Prominent interstitial damage with some foci of interstitial fibrosis was pointed out. These finding are in agreement with the inflammatory damage described.

## Relevant COVID-19 clinical aspects

Main radiological, clinical and laboratory findings are discussed below (Table 2). An intense immune response may account for alterations detectable at CT scan during severe infections. In the early phase (within 7 days from symptoms rising), numerically limited areas of ground glass opacity reflecting initial invasion of lung interstice are usually found, while ground glass opacity is often associated with repairing process signs, such as reticular pattern, vacuolar sign, fibrotic steaks, pleural involvement exc. in the advanced-phase (8–14 since symptoms rising) [5]. Severe pulmonary inflammations require oxygen supply and intensive care unit recovery.

**Table 2.** Predictive and prognostic significance of clinical findings in the course of coronavirus.

Clinical findings	Prognostic significance	Ref.
CT findings	Ground glass opacity occurs during initial pulmonary invasion; signs of interstitial damage are detectable in advances phases of infection.	[5]
RT-PCR	CT scan increases diagnostic sensitivity during the rising of infection before RT-PCR positivization and predicts infection healing before RT-PCR negativization.	[36]
Virus detection	Viral shedding lasts up to 37 days.	[37]
IL-6, lymphopenia	Most reliable and specific predictors of more severe inflammation and worse prognosis	[5,6,37]
Corticosteroids	Definite evidence about their administration is not conclusive. To date, they are demonstrated to slow viral clearance.	[38–42]

In a very large cohort of patients with suspected COVID-19, the positive rates of reverse transcriptase-polymerase chain reaction (RT-PCR) from swab samples and chest CT imaging were 59% (601/1014) and 88% (888/1014) respectively. Sensitivity of chest CT scan was predictably higher in RT-PCR+ patients (97%, 580/601). More substantially, among 308 out of 413 patients with negative RT-PCR, 48% were attested as high likely and 33% as probable cases. CT scan was indeed more sensitive in detecting initial radiological abnormalities before RT-PCR positivization and radiological regression before RT-PCR negativization [43]. We can deduce that a clinically suggestive case of SARS-CoV-2 infection with predominant respiratory symptoms should be investigated with CT scan if RT-PCR results negative. CT scan was confirmed as efficient and sensitive diagnostic tool to detect precociously inflammatory damage before symptoms arising [36].

Duration of viral shedding is a critical issue to face, especially for isolation procedures. Longest time of viral shedding was 37 days among survivors, with a median time of SARS-CoV-2 detection of 20 days, usually prolonged until death in nonsurvivors [37].

Currently, only a few laboratory markers are available to evaluate severity of COVID-19 [5,6]. Longer prothrombin time, higher D-Dimer, lower albumin, higher neutrophil count can occur in cancer patients, for instance in case of significant hepatic involvement. Higher age, higher LDH, higher cardiac troponin I, higher creatine kinase, higher serum ferritin, higher creatinine and higher procalcitonin are associated with risk of death. In absence of demonstrated link to virus-activity, they may reflect a severe organs damage in advanced phases of infection.

Coherently with inflammatory cascades previously described, lymphopenia seems to be sufficiently specific to suspect COVID-9 related severe damage and IL-6 increase was associated with increased risk of in-hospital death [37].

Use of corticosteroids (CCS) is not definitely recommended during viral pulmonary infections. Evidence about CCS treatment for COVID-19 is not definite yet [38], with the exception of singular cases in which they can play an effective role [39]. Indeed, CCS are demonstrated to delay viral clearance in pharyngeal swab and in feces, providing a rationale to avoid them in mild forms at least. Interestingly, persistent low CD4^+^ T count is associated with longer fecal RNA persistence, allowing to suppose that gastro-intestinal system is one of the main virus target and is involved in similar to lung inflammation, despite in less sever grades [40]. Not by chance, a relevant number of patients hospitalized for COVID-19 suffer from diarrhea [4,5], since ACE2 is expressed in small intestine mucosa [41].

Furthermore, CCS were not only ineffective in treating pulmonary inflammation, but they delayed RNA clearance from blood and respiratory tract and increased side effects in patients affected from similar to COVID-19 syndromes [42].

Data concerning with hepatic involvement are quite rare. Increase in aminotransferases was described among nonsurvivors compared with survivors in a large cohort [37]. In our opinion, liver injury is probably attributable to multiorgan damage observed in most severe cases.

To date, a causal treatment for COVID-19 does not exist; independent clinical trials using anti-interleukin or antiviral drugs are ongoing [44].

## Immunotherapy effects on immune system

Exact mechanisms and influences exerted by ICI are not fully understood. We provide useful insights about immunological changes potentially influencing immune response to SARS-CoV upon immunotherapy treatment (Table 3).

**Table 3.** Main effects of immunotherapy on immune cells.

Immune cells	Effects exerted by immunotherapy	Ref.
Humoral immunity	Hyperproduction of immunoglobulins	[45–47]
CD8^+^ and CD4^+^ T	Recruitment of CD4^+^ and CD8^+^ T cells typically occurs during immunotherapy treatment	[48–50]
Natural killer cells	Immunotherapy strengthens natural killer activity	[51,52]

Main approved immunotherapic drugs are anticytotoxic T lymphocyte-associated protein-4 (CTLA-4 or CD152), antiprogrammed death-ligand 1 (PD-L1, or CD274 or B7 homolog 1, B7-H1) and antiprogrammed cell death protein 1 (PD-1 or CD279) antibodies.

CTLA-4 is expressed by CD4^+^ and CD8^+^ lymphocytes. It is competitor of CD28 for T-cell co-stimulatory receptors (B7-1 or CD80 and B7-2 or CD86) during first phases of immune response [53] and inhibits T cell mediated inflammation by IL-2 suppression. IL-2 itself induces its expression on naive T cells [54], while it is constitutively expressed on forkhead box protein 3 (FoxP3)+ T_reg_ [55]. CTLA-4 thus reduces T cell activity and contributes to T_reg_-mediated immunosuppression [56].

PD-1 is expressed by many cellular phenotypes, such as B and T lymphocytes, dendritic cells, macrophages, endothelial, epithelial, muscular and trophoblastic cell [57], while PD-2 can be detected on antigen-presenting cells [58] and on activated CD4^+^ T cells [59]. The former exerts a much more important role and is broad more involved in targeting therapies than the latter.

Binding of PD-1 to PD-L1 and to PD-L2 significantly reduces T-cell proliferation and cytokines production [60,61]. PD-1 expression on naive T cells requires T cell receptor (TCR) activation [62] in presence of persistent stimulation driven by self or foreign antigens [63] and, unlike CTLA-4, it is maintained during chronic infection and cancer [64]. Even thought PD-1 expression aims at inhibiting T cell, it reflects the degree of T-cell potential activation. Both in virus-related [65] and in non virus-related cancers [66], PD-1 expressing T cells enrichment predicts better outcome upon anti-PD-1 treatment. Clonality of intratumoral PD-1+ and circulating PD-1+ T cells is quite restricted and it is tumor driven [67].

Hence, we will focus on potential shared pathways and mediators involved in immunological and inflammatory response to SARS-CoV-2 and PD-1 axis-oriented treatments, due to their far larger clinical use.

### Humoral immunity

ICI have been demonstrated to enhance humoral immunity. Blocking interaction between PD-1 and B cell PD-L1 induces not only increased clonality of circulating B cells, but also a proliferation of plasmablasts [68] and a notable immunoglobulin production [45]. Stimulation of antibodies production is the main reason why organ-specific immune-mediated inflammatory manifestations can occur upon ICI treatment [46]. PD-L1 inhibition enhances humoral immunity by modulating T_reg_ function [47]. *In vivo* experiments showed that immunotherapy increases the ratio of T_eff_/T_reg_ leading to harvested immune reaction to cancer [53].

### Cellular immunity

Restoration of lymphocytes activity during ICI usually causes a hyper-stimulation and tissue infiltration of CD8^+^ rather than CD4^+^ T cell, via IFN-γ [48], as observed in patients affected by non-small-cell lung cancer developing skin toxicity [69].

PD-1 pharmacological inhibition arises the number of T cell, B cell and myeloid-derived suppressor cells in tumors. CD8^+^ effector memory T cells are the most stimulated, above all among responders [49]. CD8^+^ T cell raising following anti-PD-1/PD-L1 interaction has been largely described, with most increase specifically in PD-1+ T cell [50].

Both viral infections and cancers provide a chronic and persistent antigenic load, among which PD-1, leading to T-cell exhaustion. Notably, blockade of PD-1 was demonstrated to promote tumor and tissue natural killer activity and antibody production indirectly or by direct effects on PD1+ B cells [51,52].

A clinical aspect to take into account is that lymphopenia occurs precociously in 70% of patients prone to develop irAE, but causal mechanisms to our knowledge are not identified yet [70].

Prevalent M2 macrophage phenotype has been described in cancers [71]. Myeloid-derived suppressor cells are immature cells with immunosuppressive effects overexpressed in cancers; they promote T_reg_ function by IL-10 and induce M2 phenotype thus reducing antitumoral activity [72]. Th1 cells play a pivotal role in inflammation promoting, by recruiting macrophages, natural killer cells and granulocytes [73].

### IL-6 & cytokines

IL-6 rises great attention in oncology, since *trans*-signaling due to soluble form of the IL-6 receptor not only accounts for more recurrent inflammation, but also enhances chemotherapy-resistance, tumor growth, metastasization and epithelial to mesenchymal transition [74–76]. Targeting IL-6 in cancer patients has been demonstrated to impact cancer-related symptoms [77] and to have minor role in cancer invasion [78]. IL-6 level has been supposed to be a measure of tumor invasiveness and immune-suppression [79].

Some cytokines (IL-2, IL-7, IL-15 and IL-21) are provided with *in vivo* and *in vitro* ability not only to promote T-cell activation, but also to upregulate PD-1 and its ligands [80]. IL-2, binding its receptor on T cells, is one of the main actors of T lymphocyte activation [81].

IFN-γ, despite well-known antiviral activity [82], contributes to PD-1 expression on macrophages [83]. Indeed, IFN-γ and TNF-α are hyper-produced by CD8^+^ T cell in response to cancer cells [84] and by T helper1 cells (Th1) with other chemokines creating a positive feedback toward CD8^+^ T-cell proliferation and tumor infiltration [73,85].

With regards of TGF-β, serum levels increase during PD-1 blockade [86].

## Conclusion: clinical implications for cancer patients treated with ICIs during SARS-COV-2 spread

Relying on the analysis of the effects from virus infection and immunotherapy on the immune system and hypothesizing potential and mutual interaction (Figure 1), conclusions for the clinical practice for patients infected with SARS-CoV-2 and treated with immunotherapy are suggested (Table 4).

**Figure 1.** Interplay and mutual effects of immunotherapy and SARS-CoV-2 infection on lymphocytes.

**Table 4.** Summary of main conclusions.

Clinical setting	Rational for potential interactions between SARS-CoV-2 infection and immunotherapy and clinical implications
Underestimation of infection prevalence	CT scan should be performed precociously in case of clinical suspect
PD-1 induction due to viral infection	Infected patients are likely to overexpress PD-1 thus becoming “hyper-immune” responders
Similar inflammatory stimuli involved	Immunotherapy and SARS-CoV-2 are likely to activate common immunological patterns thus paving the way to excessive inflammation. Oligo-clonal Ig production could account for higher macrophages activation and more severe lung injury.
Steroid treatment	Steroids may be administered in case of suspected immune-related diarrhea in absence of severe respiratory symptoms as ‘test-and-treat’ strategy.
Universal screening	Patients screening before starting immunotherapy is recommended to limit virus spread and to recognize potential ‘hyper-immune’ patients.
Long responders to ICI	It is reasonable to differ immunotherapy administration in patients with long lasting response to treatment in order to prevent contagion and to limit potential source of immunological activation during unrecognized infection.

CoV: Coronaviruses; ICI: Immune checkpoints inhibitor.

Real incidence and prevalence of SARS-CoV-2 are likely being underrated since most patients undergo infection without symptoms. Furthermore, RT-PCR of swab samples has a significant incidence of false negative, then, CT scan represents the main instrument in order to recognize as precociously as possible lung inflammation in the course of infection.

We are allowed to suppose that viral infection could increase immune-reactivity since PD-1 can be over induced by viral infection thus strengthening response to anti-PD-1/anti-PD-L1 antibodies.

Similarly to COVID-19 arising characterized by a clear CD8^+^ recruitment, immunotherapy first stimulates an increase in T cells, mainly with CD8^+^ phenotype. ICI and viral infection can likely have consequences in excessive CD8^+^ related upregulation. T_reg_ cells are involved in COVID-19 and their inhibition during immunotherapy may account for further increase in CD8^+^ hyperactivation.

Notably, ICI can induce a cytokines re-activation and some of mediators, especially interleukins, are involved in inflammatory cascade and lung injury during COVID-9. Spontaneous studies focusing on cytokines inhibition, first of all IL-6, are strongly welcomed.

Moreover, ICI increase humoral oligo-clonal response and macrophages activation. M2 phenotype is recurrent in cancers and it relates to higher invasiveness. Hyperproduction of specific IgG following SARS-CoV paves the way to more severe lung inflammation by stimulating macrophages. Inhibition of Fc receptors on macrophages might be a source of investigation for severe pneumonitis occurring in patients with COVID-19 receiving or not receiving ICI.

Differential diagnosis between COVID-19 and immune-related pneumonitis is challenging.

Clinical aspects may be helpful: COVID-19 seems to cause more frequently fever and cough, while dyspnea occurs later and correlates with severe lung damage. On the opposite, cough and dyspnea are main precocious symptoms of immune-related pneumonitis, while fever is not recurrent. To date, differential diagnosis can not rely on radiological features, while biopsy is not routinary.

Steroids represent the main instrument to treat immune-related adverse events. CCS are not recommended in the COVID-19 course and they decrease viral clearance. Since a remarkable number of patients affected from COVID-19 suffer initially from diarrhea, that is also a frequent irAE, we suppose that in absence of severe lung inflammation a ‘test-and-treat’ CCS strategy treatment is recommendable in order to reach a differential diagnosis between immune-related diarrhea and COVID-19-related diarrhea. However, high dosage CCS is not recommended in COVID-19 pneumonitis, limiting potential benefits from their administration in patients with concurrent COVID-19 and pulmonary irAE.

To our knowledge, RT-procalcitonin testing should be performed in all patients upon immunotherapy treatment or at least in patients starting immunotherapy in order to know ‘immunological background’ before ICI. Testing would be useful both to recognize potential hyper-immune patients during ICI and to limit viral spread by applying isolation.

Furthermore, ICI activity is known to be long lasting at least in responders patients that received >1-year treatments. It is plausible to differ ICI treatment during pandemic outbreak in those patients, preventing both hospital-related risk of contagion and to over activate immune response by ICI treatment.

Being aware of healthy carrier status would be surely helpful both to limit SARS-CoV-2 spread and to investigate effectively potential effects from ICI to viral infection.

A surveillance of viral shed is recommended since virus is eliminated for long period after acute phase, above all in patients receiving CCS.

## Future perspective

To date, data concerning with interactions between SARS-CoV-2 infection and immunotherapy treatment are lacking. Observational studies are required to describe outcomes of infected patients treated with ICI. Thanks to preclinical analysis of effects exerted by SARS-CoV-2 infection and immunotherapy on the immune system, we hypothesize mutual interactions and provide reasonable answers to clinical doubts concerning with ICI treatment during COVID-19 pandemic.

**Executive summary**

**Virus effects on the immune system**

- Angiotensin-converting enzyme 2 mediates viral entrance. Lower ACE2 function is associated with more severe lung inflammation and injury.
- Severe acute respiratory syndrome (SARS)-coronaviruses (CoV)-2 induces pyroptosis, mainly involving lymphocytes.
- Complement is activated by SARS-CoV-2.
- An intense production in anti-S-protein-IgG due to immune activation occurs accounting for lung injury trough macrophages activation.
- Antibodies production stimulates M2 macrophages sustaining pulmonary inflammation.
- An intense CD8^+^ and CD4^+^ T-cell recruitment occurs.

**Clinical remarkable coronavirus aspects**

- Ground glass opacity characterizes the early phase of infection, while it is associated with signs of intense inflammatory and tissue restoring signs in the advanced stages.
- CT scan increases diagnostic sensitivity and specificity in association with RT-PCR from swab samples.
- Viral shedding is not predictable since it lasts up to 37 days.
- Among clinical laboratory findings, lymphopenia and high IL-6 level are most associated with worse outcome.
- To date, benefit from corticosteroids administration is not conclusive.

**Immunotherapy effects on the immune system**

- Intense stimulation of humoral immunity, M2 macrophages, CD4^+^, CD8^+^ T cells.
- Activation of interplay between cytokines and immune cells.

**Clinical implications**

- CT scan should be performed precociously if coronavirus is clinically suspected, even when swab sample RT-PCR is negative.
- Viral infection is likely to induce programmed cell death protein 1, thus enhancing response to immune checkpoints inhibitor.
- SARS-CoV-2 and immune checkpoints inhibitor could simultaneously over activate CD8^+^ T cells and inflammatory storm.
- Steroids are not recommended for coronavirus treatment. If pulmonary and gastro-intestinal immune related event are suspected, a ‘test-and-treat’ strategy is plausible.
- Universal RT-PCR is desirable for patients upon immunotherapy treatment.
